# Intracavitary Electrocardiogram Guidance Aids Excavation of Rhythm Abnormalities in Patients with Occult Heart Disease

**DOI:** 10.1155/2021/2230383

**Published:** 2021-10-15

**Authors:** Yanli Wei, Ying Zhu, Xin Wen, Qing Rui, Wei Hu

**Affiliations:** ^1^Department of Critical Care Medicine, Affiliated Hangzhou First People's Hospital, Zhejiang University School of Medicine, Hangzhou, Zhejiang 370000, China; ^2^Department of Critical Care Medicine, The First People's Hospital of Chang Zhou, Changzhou, Jiangsu 213003, China

## Abstract

In this paper, the analysis of intracavitary electrocardiograms is used to guide the mining of abnormal cardiac rhythms in patients with hidden heart disease, and the algorithm is improved to address the data imbalance problem existing in the abnormal electrocardiogram signals, and a weight-based automatic classification algorithm for deep convolutional neural network electrocardiogram signals is proposed. By preprocessing the electrocardiogram data from the MIT-BIH arrhythmia database, the experimental dataset training algorithm model is obtained, and the algorithm model is migrated into the project. In terms of system design and implementation, by comparing the advantages and disadvantages of the electrocardiogram monitoring system platform, the overall design of the system was carried out in terms of functional and performance requirements according to the system realization goal, and a mobile platform system capable of classifying common abnormal electrocardiogram signals was developed. The system is capable of long-term monitoring and can invoke the automatic classification algorithm model of electrocardiogram signals for analysis. In this paper, the functional logic test and performance test were conducted on the main functional modules of the system. The test results show that the system can run stably and monitor electrocardiogram signals for a long time and can correctly call the deep convolutional neural network-based automatic electrocardiogram signal classification algorithm to analyze the electrocardiogram signals and achieve the requirements of displaying the electrocardiogram signal waveform, analyzing the heartbeat type, and calculating the average heart rate, which achieves the goal of real-time continuous monitoring and analysis of the electrocardiogram signals.

## 1. Introduction

According to statistics, cardiovascular disease accounts for about one-third of all deaths worldwide each year and has become the biggest threat to human health. Today, the incidence of heart disease and cardiovascular disease is increasing due to the fast pace of life and the pressure of work and life. Therefore, the prevention and diagnosis of heart disease and cardiovascular disease are particularly important [1]. Heart disease is a chronic disease and is characterized by chronic morbidity and memory onset [2]. Patients with heart disease are mobile and scattered and do not stay in one place, so they may die at some point before they can be treated. Therefore, if we can provide timely relief measures and treatment when physiological signals such as an electrocardiogram are abnormal, we can greatly reduce the mortality rate and other accidents caused by heart disease [3]. If people can check their physiological signals at any time and know their physical condition clearly according to the results obtained from the analysis of physiological signals, then they can take the initiative to prevent some heart diseases before they occur [4]. By selecting the deep convolutional neural network as the basic framework of the algorithm, the first and second points in the proposed problem can be solved well. Also, for those patients who have just finished rehabilitation surgery and returned home, it is necessary to monitor their body changes at any time, so that they can seek medical attention at any time in case of special circumstances [5]. Of course, people can also save their physiological signals so that they are not lost and can be used as an important reference for the doctor when they seek medical attention. Therefore, the ability to collect human electrocardiogram signals and analyze them automatically is essential, which will certainly promote the rapid development of medicine in the diagnosis of heart disease and cardiovascular diseases [6].

Due to the presence of noise in the collected electrocardiogram signal such as frequency interference, electromyographic interference, and baseline drift, the preprocessing stage of the electrocardiogram signal is mainly to remove the noise by filtering the electrocardiogram signal [7]. The current electrocardiogram signal noise removal methods are quite mature. Baggish et al. proposed the use of wavelet transform coefficients to determine the denoising threshold, which has a very good noise reduction effect on electrocardiogram signal denoising [8]. Hadeed et al. used IIR and FIR filters to remove the three main types of noise from electrocardiogram signals and compared the two noise removal filters. Hadeed et al. proposed an automatic classification method for arrhythmia detection by implementing a robust classifier using a neural network on a Bayesian framework [9]. Shapiro et al. classify electrocardiogram signals by proposing a method using a least-squares support vector machine, which can distinguish between normal and abnormal heartbeats [10]. Burchill propose a forward neural network-based backpropagation algorithm for cardiac arrhythmias by Artificial Neural Network (ANN) automatic classification recognition [11]. The basic level of the entire network structure consists of 11 layers. The meaning of each layer of the structure diagram will be briefly explained below. The first is the input layer, which takes an ECG signal cycle as a data sample as the input of the network; then three layers of the same structure are connected. Cuomo et al. proposed an algorithm to classify electrocardiogram arrhythmias by using Discrete Wavelet Transformation (DWT) and ANN, with a final recognition accuracy of 87.01% [12]. With the increasing capability of computers, PC-based electrocardiogram monitoring systems have been developed [9]. By sending the electrocardiogram data of the human body to the PC terminal, then the PC terminal does the preliminary analysis and diagnosis, display, and storage of electrocardiogram data locally using some electrocardiogram signal analysis algorithms and electrocardiogram signal analysis software [13]. Later, due to the rapid development of the Internet, the electrocardiogram signal collected by the PC terminal is transmitted to the cloud server and processed by some electrocardiogram signal automatic analysis algorithms, and the server returns the analysis results to the user, which not only strengthens the analysis of electrocardiogram signal but also reduces the pressure of processing in one PC terminal and speeds up the response speed [14].

Although the research on electrocardiogram monitoring systems has indeed made great progress in recent years, there are still some shortcomings. For example, the cardiac Holter machine can collect and display electrocardiogram data from the human body, but it cannot transmit and analyze them. Although the cardiac BP machine solves the problem of communication data transmission, it requires user participation, and the signal acquisition period is too short, so it can only be worn when the heart feels uncomfortable, but not when some undetectable heart rhythm abnormalities occur. Although the PC-based and Internet-based approach perfectly solves the problem of real-time monitoring and analysis of electrocardiogram signals, it is limited in application and promotion due to its lack of mobility. For example, surrounding lighting equipment and various electronic instruments are interference sources, and the frequency of such interference is mainly concentrated in 50–60 Hz. It is eliminated by designing a band notch filter or digital smoothing filter algorithm, and the frequency of the ECG signal is mainly 5–20 Hz. The research and analysis of the development of automatic electrocardiogram signal classification algorithms and the state-of-the-art electrocardiogram signal monitoring and analysis systems show that current electrocardiogram monitoring systems are not able to perform convenient and long-term monitoring of human electrocardiogram signals nor can they give real-time physiological signal analysis data. In this thesis, an improved weight-based deep convolutional neural network framework is used to study the automatic classification of electrocardiogram signals, and the algorithm model is embedded in a mobile platform to design an electrocardiogram analysis system that can perform mobile monitoring and real-time analysis of electrocardiogram signals conveniently. We analyze the current state of research on automatic electrocardiogram signal classification algorithms as well as the history of electrocardiogram monitoring systems and possible problems at various stages, propose a general plan for system design, and analyze the need for monitoring software for automatic electrocardiogram signal analysis based on a mobile platform. The basic characteristics of electrocardiogram signals are studied, and the algorithm that can correctly classify and identify electrocardiogram signals based on deep convolutional neural networks is designed and improved, and the algorithm model is saved to run on the mobile platform.

## 2. Design of Intracavitary Electrocardiogram-Guided Procedure to Assist in Mining Heart Rate Abnormalities

### 2.1. Design Analysis of Intracavitary Electrocardiogram Guidance

Abnormal heart rhythms are an important group of cardiovascular disorders [15]. There are a wide variety of cardiac rhythm abnormalities, with an irregular, rapid, or slow heartbeat. Among the more common types of heart rhythm abnormalities are the following: left bundle-branch block, right bundle-branch block, ventricular premature beats, and atrial premature beats [16]. The maximum APC weight value can be 7.8, so the corresponding normal weight value is within (0, 0.26). For the other three types of PVC, the sample size is about 4 times that of APC, so when choosing the weight value of these three categories, it is set to 1/4 of APC. The types of normal rhythms and these common types of abnormal heart rhythms will be described next. Normal rhythm is the predominant type of electrocardiogram signal, with P-wave, QRS wave, T-wave, and tiny U-wave in the waveform pattern, and occurs when there is a blocking delay or interruption in the left bundle-branch conduction system, which is a typical left bundle-branch block in the database. The incidence of these abnormalities is age-dependent, with the incidence increasing with age [17].

The S-T direction is opposite to that of the QRS main wave, and the S-T segment is elevated. On the waveform characteristics, the QRS wavelength is greater than 0.12 seconds, and the R peak is longer than or equal to 0.06 seconds. This kind of abnormality occurs when the right bundle-branch prolongation occurs, causing the right bundle-branch conduction system to suffer from blocking conduction delay or interruption. This is a typical right bundle-branch block in the database [18]. The right bundle-branch conduction block is a typical right bundle-branch block in the database [19]. The waveform pattern of the right bundle-branch conduction block reflects that the waveform before the QRS wave is relatively normal, the S wave widens and extends more downward, a small depression appears between the S and T segments, and the T wave is inverted. In terms of waveform characteristics, the QRS wave is longer than or equal to 0.12 seconds and the S wave is longer than or equal to 0.04 seconds, as shown in Figure 1.

The subjects selected for screening included both newborns and children already enrolled in school, both males and females, both urban and rural hukou populations, both cities with higher air pollution and cities with cleaner air quality, and randomly screened children with a positive diagnosis of congenital heart disease, whose screening criteria met the entry criteria for this study, since a total of 877 children with congenital heart disease were randomly screened from January 1, 2018, to December 31, 2019, and 877 children with congenital heart disease were screened for early detection of arrhythmias and follow-up for simple congenital heart disease conditions including septal defect, ventricular septal defect, unobstructed foramen oval, unobstructed ductus arteriosus, not included aortic torsion, tetralogy of Fallot, single ventricle, and other complex congenital heart disease. The abovementioned children did not have dizziness, headache, palpitations, and other symptoms before the screening of congenital heart disease (the same kind of symptoms due to the decline in cardiac function caused by congenital heart disease are not an exclusion criterion) or confirmed diagnosis of arrhythmias or hospitalization due to arrhythmias [20]. It can be found that the classification accuracy of the ECG signal after denoising processing is higher than the classification accuracy without denoising processing. The classification accuracy of the other four categories is similar, indicating that the ECG signal after denoising can improve the accuracy of the classification.

For patients with congenital heart disease who need to be hospitalized, electrocardiogram monitoring and 12-lead electrocardiogram examination were routinely performed during the hospitalization, and some patients underwent 24-hour dynamic electrocardiogram examination; for patients with abnormal electrocardiogram, they were rechecked two to three times in a week on average. For patients whose condition is not suitable for medical intervention, open thoracic surgery will be performed as the surgical group, while some patients whose condition is not suitable for surgical treatment or who have not undergone surgery for various reasons will be treated as the nonoperative group. Patients with congenital heart disease (both operated and unoperated children) who are discharged from the hospital are followed up for arrhythmias (outpatient follow-up after discharge) for about 3–12 months (average about 0.5 years).

### 2.2. Abnormal Heart Rate Design Analysis for Occult Heart Disease

The basis of abnormal heart rhythm detection lies in accurate heartbeat interception, the abnormal heartbeat on the electrocardiogram performance, that is, the appearance of more abnormal patterns.

The first step in the detection of abnormal heart rhythms is to intercept the heartbeat, splitting a section of the electrocardiogram signal into a single heartbeat, and then feature extraction of the segmented heartbeat, and then you can detect abnormal heart rhythms through machine learning. In today's social situation, as people's lives are getting faster and faster, the pressure on work and life is gradually increasing, resulting in the increasing incidence of heart disease and cardiovascular disease. If the length of the segmented heartbeats is too long, there will be a lot of data redundancy, and the accuracy of feature extraction will be affected [21]. On the other hand, if the segmented centroid is too short, some important data may be missed, which will cause errors in feature extraction. The width of the QRS wave group is known to be in the range of 0.05 s–0.l2 s, and because the data frequency in the MIT-BIH is 360 Hz, the heartbeat intercepted in this paper will be centered on the R peak, with 45 samples backward and 25 samples forward, as shown in Figure 2.

After all, subjects signed the informed consent form, intracardiac electrophysiologic study (EPS) was performed, and radiofrequency ablation was performed after the diagnosis was confirmed [22]. Intracardiac electrophysiologic measurement + ablation procedure: after the relevant surgical instruments and patients are well prepared, the patients are sterilized in the cardiac catheterization interventional room and sterile precautions such as towel laying are taken. Under local anesthesia, the left subclavian vein, left femoral vein, and right femoral vein are punctured and the 10-pole electrode catheter is placed in the coronary venous sinus (CS) area under X-ray fluoroscopy, the 4-pole electrode catheter is placed in the His bundle (HBE) area, and the 2-pole electrode catheter is placed in the right ventricle/right atrium (right ventricular, RV/right atrial, RA) in the corresponding site, adjusting the stimulation parameters to perform routine intracardiac electrophysiological examination. Through the atrial and ventricular procedures and incremental stimulation, the left and right bypasses are excluded one by one [23], and the diagnosis of AV node dual pathway can be confirmed by the presence of typical jumping phenomenon and tachycardia episodes or echoes during the procedure, followed by slow pathway improvement of the AV node [24]. When the AV node double pathway is associated with concealed conduction, it is easy to develop AV block (AVB) in the sinus rhythm state, and the etiology of this phenomenon is usually unknown, which may cause the clinician to misjudge and give incorrect treatment. If the physiological signals such as electrocardiogram (ECG) and other physiological signals are abnormal, timely relief measures and treatment can be provided, which can greatly reduce the mortality and other accidents caused by heart disease. There have been reports of patients who were misdiagnosed as having AVB in the clinical diagnosis and had a permanent pacemaker implanted. Pacemaker implantation due to misdiagnosis is often associated with unforeseen risks, such as intraoperative bleeding, postoperative infection, and even complications such as irreversible cardiac rupture. The clinical and electrophysiological characteristics of the 11 patients included in this paper were observed and followed up to analyze the factors associated with AVB.

The MIT-BIH arrhythmia database is the most authoritative and extensive database for the study of arrhythmias and is provided by the Massachusetts Institute of Technology (MIT). Electrocardiogram data were from individuals, 47 of whom consisted of 25 males and 22 females, for a total of 48 recordings (data 201 and 202 were taken from the same male individual). These 48 records were sampled at a frequency of 360 HZ, in two leads, for approximately 30 minutes. Each record is annotated by more than two electrocardiogram experts, and each beat cycle of electrocardiogram signal is analyzed, independently annotated, and then verified and reviewed, and the rhythm type of electrocardiogram signal is decided by final consensus. The arrhythmia database is used as an authority to study abnormal heart rhythm data. The correspondence between the annotation information of MIT-BIH is shown in Table 1.

Through the investigation and analysis of the requirements of the common abnormal electrocardiogram signal mobile platform analysis system, including the whole process from the acquisition of the electrocardiogram signal, through the Bluetooth transmission to the end for analysis and the result visualization, this paper determines the direction and goal of the whole system implementation. Although the PC-based and Internet-based methods perfectly solve the problem of real-time monitoring and analysis of ECG signals, because they are not mobile, they will be greatly restricted in application and promotion. The monitored person is connected to the electrocardiogram acquisition terminal through the way of three leads, collecting the human body's electrocardiogram signal, sending the data through Bluetooth module after signal processing means, and receiving the human body's electrocardiogram data through Bluetooth in real time in the client. Analysis and the results of the analysis determine the need to alarm the relevant personnel. The monitored personnel will be able to view their physiological health status in real time through the client.

According to the data flow diagram of the system, the main functional requirements of the system are electrocardiogram data collection and transmission, electrocardiogram data reception, and real-time electrocardiogram display, electrocardiogram signal waveform detection, automatic analysis, alarm judgment, and electrocardiogram data preservation and management.

### 2.3. Evaluation Index Design Analysis

In the MIT-BIH arrhythmia database, 75.25% of the electrocardiogram signals are normal electrocardiogram signal types, while the four abnormal signal types account for only about 24.75%. Therefore, an imbalance problem arises in the data processed in the MIT-BIH arrhythmia database. The so-called data imbalance problem refers to the highly skewed distribution of the classification samples. In this paper, the normal type is much more than the other four types of abnormal electrocardiogram signals, which will cause a large error in the classification of abnormal electrocardiogram signals. How to improve the algorithm framework for data imbalance is the most important issue in the algorithm design process, which is the main improvement of the algorithm in this paper.

From the above analysis, deep convolutional neural networks can be carried out together with sample feature extraction and classification identification in the classification identification process. When transplanted to the platform, the developer only needs to care about the input and output of the model, and the work of intermediate waveform localization and feature extraction can be eliminated, minus the complexity caused by the transplantation of the algorithm model, so the deep convolutional neural network as an algorithm framework can be conveniently applied in the platform. By choosing a deep convolutional neural network as the algorithm framework, the first and second points of the proposed problem can be well solved. For the third point of data imbalance problem, the basic deep convolutional neural network framework cannot solve such problems, so the algorithm framework needs to be improved, as shown in Figure 3.

After the above specific analysis of each level, analyzing the characteristics of each level in the deep convolutional neural network and the abnormal electrocardiogram signal classification problem to be solved in this paper and the specific hierarchical structure of the input and output layers as well as the intermediate basic levels of convolutional, pooling, and fully connected layers are determined. As shown in Figure 4, the basic network structure of the deep convolutional neural network electrocardiogram signal classification algorithm is proposed in this paper, and the whole network structure contains 11 layers. Study the basic characteristics of the ECG signal, according to the characteristics of the deep convolutional neural network, design and improve the algorithm that can correctly classify and recognize the ECG signal, and save it as an algorithm model running on the mobile platform. The first layer is the input layer, which takes an electrocardiogram signal period as a data sample as the input of the network; then it is followed by three similar layers, which include a convolutional layer, a convolutional block composed of a convolutional layer, a normalization process, and an excitation function Rely, and a pooling layer, which can complete the extraction of electrocardiogram signal features and avoid inaccurate waveform localization and artificial selection. The errors of the eigenvalues are then connected to three fully connected layers to map the eigenvectors to the labels, and the final output layer is used to obtain the output results of the five heart rhythm types.

## 3. Results and Analysis

### 3.1. Analysis of Experimental Data Processing Results

This system enables automatic analysis of electrocardiogram signals by using a convolutional neural network model framework. However, training the network model requires a large number of data samples, i.e., the input of the network, and there are two ways to obtain the general deep learning dataset: the first one can use the public dataset on the Internet, which eliminates the steps of dataset processing, and the second one is that the data is publicly available on the Internet or there is no corresponding dataset, which requires manual hands-on production of the dataset. The MIT-BIH database contains 60 groups of signals with a sampling frequency of 360 Hz, and each group of signals is sampled continuously for nearly 32 minutes. Figure 4 shows a continuous waveform of the electrocardiogram signal from the intercepted MIT-BIH database 101 data, but the doctor's analysis of the electrocardiogram is based on one heartbeat, so the electrocardiogram signal is divided into one heartbeat. Therefore, although there are 48 sets of MIT-BIH arrhythmia data, they still cannot be used as the input of the convolutional neural network model, so we need to preprocess the 48 sets of data first, and the preprocessing process mainly includes MIT-BIH data parsing, electrocardiogram signal denoising, and beat division.

The first line of the record represents the record as data number 101, which contains two signals and the sampling frequency is 360 Hz with 650,000 sampling points. In the waveform shape, there are P-wave, QRS wave, T-wave, and tiny U-wave in sequence. This kind of abnormality occurs when there is a delay or interruption of block conduction in the left bundle-branch conduction system, which is a typical left beam of the database. The next two lines record information for two sets of signals, respectively, which represent data number 101 and are stored in the “212” mode. 200 refers to the ADC gain, 11 refers to the ADC resolution, the ADC zero value is set to 1024, and the first value of the sampled signal is 955. And the next two large integers indicate the number of checks that were performed on the sampling sites. The fourth-row records patient information, with age, gender, and record data, respectively. The last row records the patient's medication history.

In the MIT-BIH record reading process, each record is firstly read as a file, and then the parameters of each record are parsed according to the previous record format; after the format parsing, the MLII channel of the two groups of signals is selected, and then all the original records are read according to “212” format, including atrial septal defect, ventricular septal defect, patent foramen oval, and patent ductus arteriosus. After getting the record-sampled raw data, the next step is to denoise the electrocardiogram signal for each record. However, considering the special characteristics of the convolutional neural network, the data samples can be directly inputted into the network without denoising, and the network also has a certain denoising effect, so this paper divides two data sets on whether the electrocardiogram signal is denoised or not and carries out the simulation experiments respectively, as shown in Figure 5.

The frequency distribution of the main components is between 20Hz and 5000Hz. power frequency interference is a common interference in the power network; for example, surrounding lighting equipment and a variety of electronic devices are interference sources, and such interference frequency is mainly concentrated in the 50–60 Hz. Through the design of a band trap filter or digital smoothing filter algorithm, the elimination was performed, while the cardiac signal frequency was mainly in the range of 5–20 Hz.

After determining the specific steps of the heartbeat division method, the two groups of data use this method to divide the heartbeat separately to obtain two data sets. First of all, the 48 groups of data without denoising are divided into five categories, and the corresponding heartbeats are placed in one category to obtain the data set Set1; similarly, the 48 groups of data after denoising are divided to obtain the data set Set2; the final results of the two data sets are shown in Figure 6.

The experimental data taken in this paper is from the MIT-BIH arrhythmia database; in the experimental data processing step, the data from the database has been converted into the input of the network, followed by the simulation experiments, and the results of the model simulation experiments are analyzed and discussed (Figure 7).

In this paper, the algorithmic framework without adding weights is used as the improvement algorithmic model, but the network, which will be improved according to the improvement strategy, will be used as a deep convolutional neural network based on weights, i.e., the improved algorithmic model. The original dataset Set1 is now used as the experimental data to perform the experiments separately. Before conducting the experiments, we need to set the weights of the improved deep convolutional network model Cross-Entropy first.

Firstly, since the sample size of Normal is about 30 times that of APC, the corresponding weight of Normal is set to 1/30 of APC, and the maximum APC weight is 7.8, so the corresponding weight of Normal is in the range of (0,0.26). For the other three types of RBBBB, LBBBB, and PVC, the sample size is about 4 times the APC sample size, so the weight of these three types is set to 1/4 of the APC, and according to the determined Normal weight range, the step size is 0.02, and the weight with the highest accuracy is the final weight.

### 3.2. Analysis of Excavation Results

According to the specific idea of weight setting, take the step length of 0.02 and perform the experiment in the range of (0, 0.26), and the specific experimental results are shown in Figure 8, where the horizontal axis represents the Normal weight setting value and the vertical axis represents the overall accuracy of the network model.

After the experiment, it is found that the overall accuracy is the highest when the Normal weight is set to 0.2, so the final Normal-type weight is set to 0.2, each type is calculated according to the idea of weight setting, and the final weight setting value is shown in Figure 8.

The datasets all use the original dataset Set1, and the two network models keep the same parameters except for the difference in the Cross-Entropy weights. The network learning rate is set to 0.001 and the number of learning iterations is set to 250.  Figure 9 shows the overall accuracy of the network model before and after the 250 iterations, and Figure 9 shows the loss of the network model before and after the 250 iterations.

From Figure 9, we can see that the overall accuracy of the improved network model is significantly higher than the curve before the improvement, which is better than before; from Figure 9, we can see that the loss before the improvement is above 0.01, and the loss after the improvement is down to about 0.001, which is much lower than the model loss. Some of the patients underwent 24-hour dynamic electrocardiogram examination. For those with abnormal electrocardiogram, reexamination was performed 2 to 3 times in an average of 1 week. However, these two figures can only show that the overall classification identification rate of the network model with increased weights is better than before, but this paper is mainly concerned with the classification and identification accuracy of the four types of abnormal electrocardiogram signals, so the following is the specific classification of each type of situation and evaluation index results.

The main content of the test is the test of the data receiving module and the overall system function module. The data receiving module test is mainly Bluetooth pairing connection test, and data parsing processing test, to ensure the correctness and integrity of the received data. After a series of testing and debugging, the overall system function can be stable and run for a long time.

In the experimental data processing stage, two data sets, Set1 and Set2, were made according to whether to denoise the electrocardiogram signal data. The network model results for the original dataset Set1 are shown in Figure 10, and the following experiments are conducted on the denoised dataset Set2 using the improved model. The experimental classification results are shown in Figure 10, where the vertical axis represents the actual heartbeat type and the horizontal axis represents the model prediction results. The results of the classification evaluation metrics are shown in Figure 10.

From Figure 10, it can be seen that the experimental results of the algorithmic network model for the denoised data set Set2 are all above 95% except for the APC type, and although the recognition rate of the APC type does not reach the same as the other types, it is also improved compared to the data before denoising. Comparing the data set after denoising with the data set without denoising, there is a small improvement in all three indicators of APC type, but the improvement is not significant for the other four types because the APC type is like Normal-type in waveform morphology. The reason the classification accuracy is still so high is that the number of normal heartbeats accounts for a very large proportion of the dataset, thus the classification accuracy can be maintained at a relatively high level. Comparing the simulation results of Set1 and Set2, it is found that the classification accuracy of the denoised electrocardiogram signal is improved for APC types compared with that of the nondenoised one, and the classification accuracies of the other four types are similar, indicating that the denoised electrocardiogram signal can improve the recognition accuracy of APC types and will not affect the classification of the other types. Therefore, in this paper, denoising is firstly performed on the collected electrocardiogram signal, and then the classification and identification are performed on the denoised electrocardiogram signal.

## 4. Conclusion

This paper fully investigated the research content and research status of common abnormal electrocardiogram signals, summarized some algorithms in the automatic classification of electrocardiogram signals, elaborated on the specific measures taken by these traditional classification algorithms in the process of automatic classification of electrocardiogram signals as well as their shortcomings, and determined the research ideas and relevant technical theoretical knowledge. Besides, for the electrocardiogram signal mobile platform analysis system, the development history of the electrocardiogram monitoring system is analyzed, and the direction and goal of the mobile platform analysis system are determined in this paper after analysis and comparison. The functional and performance requirements of the mobile platform system for common abnormal electrocardiogram signals were designed, and the functional modules and the links between them were identified. To address the shortcomings of traditional electrocardiogram signal classification algorithms and their inconvenience in engineering applications, this paper proposes a weight-based deep convolutional neural network as a framework for electrocardiogram signal classification algorithms, which eliminates the need for manual feature extraction, reduces the complexity of the algorithm, and can be deployed quickly and invoked on the end. Two datasets were constructed using data from the public database MIT-BIH, and the classification results of the two datasets were compared to finalize the process of denoising the electrocardiogram signals before analyzing and processing them.

## Figures and Tables

**Figure 1:** Intracavitary electrocardiogram guidance design framework.

**Figure 2:** Heartbeat interception diagram.

**Figure 3:** Evaluation process design.

**Figure 4:** Schematic diagram of a continuous segment of the electrocardiogram signal.

**Figure 5:** Simulation experiment results.

**Figure 6:** Five types of results.

**Figure 7:** Setting range of weights.

**Figure 8:** Experimental results of weight setting.

**Figure 9:** Comparison of the overall accuracy change of the network model before and after improvement.

**Figure 10:** Identification results.

**Table 1:** MIT-BIH annotation code correspondence table.

Comment code	Symbol	Remarks	Values
0	—	Normal beating	3
1	L	Left bundle-branch block	3
2	R	Right bundle-branch block	3
3	a	Abnormal atrial premature beats	4
4	V	Ventricular premature beats	4
5	F	Ventricular fusion heartbeat	3
6	J	Borderline premature beats	2
7	S	Atrial premature beats	2
9	g	Supraventricular premature contractions or abnormalities	3
10	j	Ventricular escape	3
11	1	Borderline escape	2
12	—	Heartbeat	4
13	L	Uncategorized heartbeat	2

## Data Availability

The data used to support the findings of this study are available from the corresponding author upon request.
